The article "Molecular Polymorphisms of Vascular Endothelial Growth Factor Gene and Bronchopulmonary Dysplasia in Very Low Birth Weight Infants" was published in 2022. Journal: Dis Markers.

# Molecular Polymorphisms of Vascular Endothelial Growth Factor Gene and Bronchopulmonary Dysplasia in Very Low Birth Weight Infants

**DOI:** 10.1155/2022/2793846

**Published:** 2022-09-01

**Authors:** Laura Filonzi, Serafina Perrone, Maria Luisa Tataranno, Cinzia Magnani, Harold Dadomo, Anthea Bottoni, Marina Vaghi, Francesco Nonnis Marzano

**Affiliations:** ^1^Department of Chemistry, Life Sciences and Environmental Sustainability, University of Parma, Italy; ^2^Neonatology Unit, University Medical Center of Parma (AOUP) and University of Parma, Parma, Italy; ^3^Neonatology Unit, University Medical Center Utrecht and Utrecht University, Utrecht, Netherlands

## Abstract

**Background:**

Bronchopulmonary dysplasia (BPD) is a chronic lung disease affecting primarily preterm and very low birth weight (VLBW) infants. Despite the advances in perinatal care, BPD remains a major clinical and costly complication in premature infants. The pathogenesis of BPD is complex and multifactorial. Prematurity, mechanical ventilation, oxidative stress, and inflammation are recognized as major interrelated contributing factors. Recently, some candidate genes involved in angiogenesis and alveolarization regulating mechanisms have been associated to BPD risk development. The aim of this study was to evaluate the role of vascular endothelial growth factor (VEGF) polymorphisms on BPD onset in VLBW newborns.

**Methods:**

Eighty-two VLBW infants, without major anomalies, were consecutively enrolled: 33 developed BPD (BPD group) and 49 infants without BPD served as controls (control group). In all infants, two polymorphisms, respectively (VEGF receptor) *VEGFR1*-710 C/T and *VEGF* +936 C/T, were determined through salivary brush. Genomic DNA was extracted and purified from saliva samples by using the MasterAmp Buccal Swab DNA Extraction Kit (Tebu-bio, Milan, Italy).

**Results:**

Significant statistic differences were found between BPD newborns and controls with regard to gestational age, birth weight, mechanical ventilation, duration of oxygen therapy, maternal preeclampsia, and chorioamnionitis. No differences were detected between genotypic and allelic levels regarding *VEGFR1* and *VEGF* molecular polymorphisms.

**Conclusions:**

Two single nucleotide polymorphisms within *VEGF* and *VEGFR1* genes are not associated with BPD. Further researches are needed to reveal gene polymorphisms involved in vascular development as contributors to the onset of BPD.

## 1. Introduction

Bronchopulmonary dysplasia (BPD) is considered to be the most common cause of pulmonary morbidity in very preterm infants. It is associated with life-long morbidities and remains one of the most serious and difficult challenges in very preterm infant care. Although survival of extremely preterm infants (below 28 weeks of gestational age (GA)) has increased over the past 2 decades, the rate of BPD still ranges from 40% to 55% among infants of 26-27 weeks [1]. BPD can be defined as requirement of additional O2 at 36-week postmenstrual age (PMA) [2]. Pathogenesis of BPD has been recognized as multifactorial [3].

The article "Molecular Polymorphisms of Vascular Endothelial Growth Factor Gene and Bronchopulmonary Dysplasia in Very Low Birth Weight Infants" was published in 2022. Journal: Dis Markers.

In addition to clinical factors, evidence from twin studies suggested a genetic predisposition to determine the development of BPD [4].

Several candidate genes that affect BPD-associated biological pathways has been identified by a genome wide association study [5].

Current (new) BPD is characterized by large simplified alveolar structure, reduced and dysmorphic vascular bed with rare epithelial lesions, and mild airway smooth muscle thickening [6].

The vascular endothelial growth factor (VEGF) is a relatively specific endothelial cell mitogen that regulates angiogenesis and endothelial cell differentiation. It is a key regulator of vascular repair and of alveolar growth in the developing lung. VEGF has multiple roles in vascular development and maintenance and is essential for the formation of embryonic vasculature [7, 8]. Previous studies have shown that VEGF inhibition during the early neonatal period determines alveolar and pulmonary vascular structure chronic abnormalities, which are characteristic of pathological changes in human BPD [9–12].

The *VEGF* gene is located on chromosome 6 (6p21.3) [13] and consists of 8 exons. Several polymorphisms of *VEGF* such as +936 C/T, -2578 C/A, -406 C/T, and -1154 G/A have been identified and have been associated with VEGF protein production variations [14–16]. Among them, the *VEGF* +936 C/T polymorphism (rs3025039) is the most widely studied [17]. Soluble vascular endothelial growth factor receptor 1 (VEGFR1) is one of the important receptors of VEGF angiogenesis signaling and plays a key role in normal vessels formation processes. VEGF was found decreased in tracheal fluid samples in preterm newborns who subsequently developed BPD, and lung VEGF and VEGF receptor 1 (VEGFR1) expressions were found decreased in infants who died following BPD [12]. Moreover, Tang et al. [11] suggested that damaged VEGF signaling in utero interrupts lung growth and contributes to the increased risk of BPD.

The aim of this study was to investigate the genotypic and allelic frequencies of *VEGF* and *VEGFR1* gene polymorphisms in VLBW infants who developed BPD, compared to pair controls. We tested the hypothesis that alleles encoding the less efficient isoforms would have increased frequency in the BPD population.

The article "Molecular Polymorphisms of Vascular Endothelial Growth Factor Gene and Bronchopulmonary Dysplasia in Very Low Birth Weight Infants" was published in 2022. Journal: Dis Markers.

## 2. Patients and Methods

A prospective study was conducted in the Neonatal Unit of Parma University Hospital in a period of five years. The study was approved by local Ethical Committee (Protocol Number 45428). Written informed consent was obtained by parents of enrolled population. Patient recruitment criteria were (1) preterm birth less than 32-week gestational age and (2) birth weight less than 1500 g (VLBW). Infants with major anomalies and without informed consent from the parents were excluded from the study.

BPD patients were defined as follows: the need of O2 supplementation at 36 weeks of gestational age.

Detailed perinatal data (birth weight, gestational age, Apgar score at 1 and 5 minutes after birth, gender, prenatal corticosteroid therapy, causes of premature deliver, need of mechanical ventilation, mode of ventilation, duration of oxygen therapy, surfactant treatment, diuretic therapy, and patent ductus arteriosus) were recorded on NICU admission.

Salivary brushes were used to collect DNA samples from buccal leucocytes. Genomic DNA was extracted and purified from saliva samples by using the MasterAmp Buccal Swab DNA Extraction Kit (Tebu-bio, Milan, Italy).

One polymorphism was selected in the promoter region of *VEGFR1* gene (-710 C/T), and another variant defined +936 C/T (rs3025039) was selected in the 3′UTR polymorphism *VEGF* gene.

The *VEGFR1* gene (-710 C/T) polymorphism was detected with the PCR-RFLP method. PCR (thermal cycler MJ Research PTC100MJ, Waltham, MA) was performed using specific primers and conditions suggested by Rodrigues et al. [17]. Following PCR, the entire sample was digested with 5 units of *Nla*III at 37°C overnight. Digested products were separated by electrophoresis on a 2.5% agarose gel. Two variants were obtained: a restricted polymorphism displayed by two fragments of 518 and 147 bp, respectively, and another one resulted in an uncut 665 bp fragment. The *VEGF* 936C/T polymorphism was analyzed using the following primers: 5′-AAG GAA GAG GAG ACT CTG CGC AGA GC-3′ (forward) and 5′-TAA ATG TAT GTA TGT GGGTGG GTG TGT CTA CAG-3′ (reverse) suggested by Traina et al. [18]. The cycling condition were 95°C 10 min, followed by 35 cycles of 95°C 45 s, 64°C 45 s, 72°C 45 s, and then 72°C 10 min. PCR amplicons were digested with the restriction endonuclease *Nla*III (New England Biolabs) for 16 h at 37°C. The 936C allele remained uncut (208 bp), while the 936T variant resulted in two different fragments of 122 bp and 86 bp, respectively [19].

### 2.1. Statistical Analyses

Statistical analyses were performed by using Statistica software (version 8.0) by StatSoft Inc. (Tulsa, OK). To investigate possible associations between genotypes/alleles and case groups, a likelihood ratio (LR) chi-square test was performed. In addition, the Yates correction was applied to the chi-square test considering the limited number of analyzed patients. An additional percentage of 20% of analyses was randomly repeated to verify data reproducibility, and no discrepancies were observed. Gestational ages, birth weight, and Apgar score, due to the normal distribution of data, were analyzed with ANOVA.

The article "Molecular Polymorphisms of Vascular Endothelial Growth Factor Gene and Bronchopulmonary Dysplasia in Very Low Birth Weight Infants" was published in 2022. Journal: Dis Markers.

## 3. Results

Eighty-two consecutive newborns were included in the study, 33 BPD infants and 49 controls (perinatal characteristics of study population are reported in Table 1). The BPD was more frequent in male newborns (20 males vs. 13 females) with a frequency of 60.6%; in contrast, the control group displayed a 48.9% frequency (24 males vs. 25 females). In the majority of pregnancies, causes of premature delivery in the case group were preeclampsia (PE) (30.3%), premature rupture of membranes (Pprom) (39.3%), and chorioamnionitis (CA) (18.1%). In the control group, the cause of premature delivery were other (Pprom 32.6%, PE 18.3%, and CA 12.2%).

Thirteen newborns (39.3%) with BPD had patent ductus arteriosus (PDA) as premature complication versus one newborn (2.0%) of the control group.

The gestational age and birth weight were significantly lower in BPD neonates with respect to the control group (Table 2). Notably, the birth weight was less than 1000 grams in 25 neonates (75.7%) of the BPD group and only in 4 control group neonates (8.2%) as reported in Table 1.

Mean value of Apgar score < 5 at 1^st^ minute and <7 at 5^th^ minute is reported in Table 2. More precisely, 66.6% of BPD neonates displayed an Apgar score 1′ < 5 and 5′ < 7 which was threefold higher than control cases (22.4%). This result was statistically supported by significant *p* < 0.00001.

As many as 30 newborns of the case group (90.9%) required mechanical ventilation during the first 3 days of life with respect to 44.8% of the control group. In BPD neonates, mechanical ventilation lasted significantly more days with respect to controls (*p* < 0.000001).

Twenty-two (66.6%) newborns received surfactant treatment in the case group, and instead, 12 (24.4%) received surfactant therapy in the control group. Twelve mothers (36.3%) received antenatal steroids in the case group and 21 (42.8%) in the control group.

### 3.1. Genetic Analysis

Concerning genetic analysis, genotypes and allelic frequencies of the *VEGFR1*-710C/T polymorphism are shown in Table 3. Although C and T alleles were detected in all considered samples, and no difference in the distribution was observed between pathologic and nonpathologic samples. Genotyping frequency of the *VEGFR1*-710C/T polymorphism was similar in all groups. In particular, 31 CC homozygote genotypes and 2 CT heterozygotes were detected in the investigated BPD infants; 46 homozygote CC genotypes and 3 CT heterozygotes were found in the control group. Interestingly, no infant affected by BPD or controls showed the TT genotype. The frequency of the CC genotype was similar in BPD cases (93.9%) and in the controls (93.8%), and the frequency of the CT genotype too (6.1% BPD vs. 6.2% controls). The C allele was found in the same percentage (96.9%) both in BPD and controls; T frequency was the same in healthy controls (3.1%) and BPD patients.

The article "Molecular Polymorphisms of Vascular Endothelial Growth Factor Gene and Bronchopulmonary Dysplasia in Very Low Birth Weight Infants" was published in 2022. Journal: Dis Markers.

Considering overall data of *VEGFR1* polymorphism, no statistical significance emerged between pathologic and control samples both at genotypic and allelic level.

Data on genotype and allele frequencies of *VEGF* 936 C/T polymorphism are reported in Table 4. No differences emerged in genetic data between the pathologic and control groups. Genotypic frequencies in BPD infants were 72.7% (CC homozygotes), 24.3% (CT heterozygotes), and 3% (TT homozygotes); in the control group, they were, respectively, 69.4% (CC genotype), 28.5% (CT), and 2.1% (TT). Considering allelic frequencies, the C allele was present in 84.8% of BPD infants and in 83.7% of the control group. There was no statistical difference for this gene between BPD patients and controls in either genotype (*p* = 0.68) or allele (*p* = 0.76) frequencies.

## 4. Discussion

Bronchopulmonary dysplasia (BPD) is a chronic lung disease in infants born extremely preterm, characterized by a prolonged need for supplemental oxygen or positive pressure ventilation beyond 36-week postmenstrual age. According to recent guidelines, BPD is present when an infant requires oxygen therapy at the age of 28 days [20]. BPD affects about 20–30% of very low birth weight infants and is a major cause of morbidity and mortality in this vulnerable population [21].

In addition, literature data showed that, besides clinical factors, a genetic predisposition could determine the development of BPD [3]. Several studies suggested that endothelial-epithelial cross-talk, especially via VEGF signaling, is critical for normal lung growth following birth and that disruption of VEGF signaling impairs lung vascular growth and alveolarization [9–12].

In this study, we sought to identify epidemiological and genetic risk factors related to vascular growth and alveolarization, contributing to the development of BPD.

From our results, it emerged that BPD incidence in our group was 29% of preterms. The major clinical risk factors for BPD in our population were premature birth (gestational age between 23 and 27 weeks) and very low birth weight (less than 1000 g), as widely expressed in literature [22, 23]. Among maternal risk factors, preeclampsia and chorioamnionitis were found significantly associated with BPD, as previously demonstrated [24–26]. Moreover, in accordance with Carey et al. [27], BPD was more frequent in male newborns rather than in females. Other important predictive factors were Apgar score and mechanical ventilation, lasting more than 3 days after birth. Patent ductus arteriosus affected more frequently newborns with bronchopulmonary dysplasia, as evidenced by the EPICE study [28].

The article "Molecular Polymorphisms of Vascular Endothelial Growth Factor Gene and Bronchopulmonary Dysplasia in Very Low Birth Weight Infants" was published in 2022. Journal: Dis Markers.

In our study, there was not a significant difference in the group of newborns who had received antenatal steroids in accordance with literature data [29, 30].

The importance of these risk factors determined in our work was already known and well described in literature.

Nowadays, genetic factors come in the focus of interest. That is why in the present study, we also focused our attention on the direct association between molecular polymorphisms and BPD, investigating genetic factors that may directly be associated with BPD development. Therefore, we evaluated one *VEGF* polymorphism (+936 C/T) and one polymorphism at the promoter of *VEGFR1* (-710 C/T). In this paper, we demonstrated no direct association between *VEGF* +936 C/T and *VEGFR1*-710 C/T gene variants and BPD, both at genotypic and allelic levels. Previous studies suggested an association between some *VEGF* polymorphisms and BPD. Mailaparambil et al. [31], considering 155 preterm newborns, found an association between rs699947 *VEGF* and BPD. A link between a *VEGF* polymorphism and BPD was described in the Polish population few years ago; in addition, Kwinta et al. [32] found an association between BPD and the VEGF -460T>C polymorphism. In relation to this, they demonstrated that VEGF -460CC homozygotes were at a lower risk than babies with -460TT or -460TC genotypes.

These discrepancies between our genetic results and those reported by other studies [31, 32] could be explained by different single nucleotide polymorphisms (SNPs) within *VEGF* and *VEGFR1* genes that we analyzed. As suggested by Bokodi et al. [20], several results concerning the association between genetic polymorphisms and BPD risk factors are negative, in spite of the known role of encoded protein in this disease pathogenesis.

These findings support the hypothesis that BPD is a heterogeneous disease that results from multiple genes and pathways. Accordingly, the two genes herein examined are not the only one that could be implicated in BPD development. Many other pathways (inflammation, anti-inflammation, airway branching, etc.) with several genes coding for cytokines, adhesion molecules, and defense antioxidant proteins are supposed to be involved [20].

The article "Molecular Polymorphisms of Vascular Endothelial Growth Factor Gene and Bronchopulmonary Dysplasia in Very Low Birth Weight Infants" was published in 2022. Journal: Dis Markers.

The small sample size may have influenced our results and the lack of genetic differences between the two groups, and it is thus a limit of this study. Although this is a preliminary report, the scarcity of data on BPD infants makes these limited cases interesting to the scientific scenery. It is noticeable that to really exclude any genetic influence, this study should have been performed in a larger population over a shorter period of time.

## 5. Conclusions

No genetic association exists between two single nucleotide polymorphisms within *VEGF* and *VEGFR1* genes and BPD onset. Further studies are needed to verify the debated role of genes involved in angiogenesis and alveolarization regulating mechanisms in the development of chronic lung diseases among very low birth weight infants.

## Figures and Tables

**Table 1:** Clinical characteristics of study population.

	Controls		BPD		*p*
	*n*	%	*n*	%	
*n*	49		33		—
Gender (male/female)	24/25	48.9%	20/13	60.6%	0.29
Patients with birth weight < 1000 g	4	8.1%	25	75.7%	0.00001
Apgar score (<5 at 1 min and <7 at 5 min)	11	22.4%	22	66.6%	0.00001
Preeclampsia (PE)	9	18.3%	10	30.3%	0.18
Premature rupture of membranes (Pprom)	16	32.6%	13	39.3%	0.53
Chorioamnionitis (CA)	6	12.2%	6	18.1%	0.39
Patent ductus arteriosus (PDA)	1	2.0%	12	36.3%	0.00001
Mechanical ventilation during the first 3 days of life	22	44.8%	30	90.9%	0.00001
Nasal continuous positive pressure (ncPAP)	22	44.8%	22	66.6%	0.0523
Synchronized intermittent mechanical ventilation (SIMV)	10	20.4%	22	66.6%	0.00001
Surfactant therapy	12	24.4%	22	66.6%	0.00001
Diuretic therapy	0	—	18	54.5%	—
Antenatal steroid treatment in mother	21	42.8%	12	36.3%	0.49

**Table 2:** Differences in gestational age, birth weight, and Apgar score between BPD group and controls.

	Controls (mean ± SD)	BPD (mean ± SD)	*p*
Gestational age (wks)	30.56 ± 0.35	28.43 ± 0.43	<0.00001
Weight (g)	1198.94 ± 140.34	895.85 ± 198.98	<0.0000001
Apgar score 1 min	6.75 ± 1.51	5.38 ± 1.43	<0.0005
Apgar score 5 min	8.33 ± 0.71	7.48 ± 0.85	<0.00005

**Table 3:** Frequencies of *VEGFR1* genotypes and alleles determined in BPD patients and controls with enclosed statistical elaboration.

*VEGFR1*-710 C/T	BPD (*n* = 33)		Controls (*n* = 49)		LR *Χ*^2^ test	*p* value
	Number	Percentage	Number	Percentage		
*Genotypes*					0.07	0.79
CC	31	93.9	46	93.8		
CT	2	6.1	3	6.2		
TT	0	0.0	0	0.0		
*Alleles*						
C	64	96.9	95	96.9	0.07	0.79
T	2	3.1	3	3.1		

**Table 4:** Frequencies of *VEGF* (936 C/T) genotypes and alleles with corresponding statistical elaborations determined in BPD patients and control group.

*VEGF* 936 C/T	BPD (*n* = 33)		Controls (*n* = 49)		LR *Χ*^2^ test	*p* value
	Number	Percentage	Number	Percentage		
*Genotypes*					0.17	0.68
CC	24	72.7	34	69.4		
CT	8	24.3	14	28.5		
TT	1	3	1	2.1		
*Alleles*					0.09	0.76
C	56	84.8	82	83.7		
T	10	15.2	16	16.3		

The article "Molecular Polymorphisms of Vascular Endothelial Growth Factor Gene and Bronchopulmonary Dysplasia in Very Low Birth Weight Infants" was published in 2022. Journal: Dis Markers.

## Data Availability

Data will be available upon request.
